# Abscopal Effect in a Patient With Metastatic Melanoma Receiving Hypofractionated Radiation Therapy and Dual Immune Checkpoint Inhibition: A Case Report

**DOI:** 10.7759/cureus.74662

**Published:** 2024-11-28

**Authors:** Jenna R Rocchetti, Jeremy Price

**Affiliations:** 1 Radiation Oncology, Rowan-Virtua School of Osteopathic Medicine, Stratford, USA; 2 Radiation Oncology, Fox Chase Cancer Center, Temple University Hospital, Philadelphia, USA

**Keywords:** abscopal effect, hypofractionated palliative radiation therapy, immune checkpoint inhibitor, ipilimumab, metastatic melanoma, nivolumab

## Abstract

Concurrent with the increasing utilization of immune checkpoint inhibitors (ICIs) in melanoma, there has been renewed interest in understanding the potential interplay between radiation therapy (RT) and the immune system. One such phenomenon is the abscopal effect, where localized treatments, such as RT, not only shrink the targeted tumor but also induce shrinkage of untreated tumors elsewhere in the body. Here, we report a case of an abscopal effect in a 63-year-old patient with metastatic melanoma who was progressing on first-line dual ICI therapy but experienced a rapid and durable systemic response following the administration of hypofractionated palliative RT to a large primary melanoma skin tumor.

## Introduction

Melanoma is the fifth most common cancer in the United States, accounting for 1.7% of global cancer diagnoses [1]. Despite representing only 1% of all cutaneous malignancies, melanoma is responsible for 80% of skin-related deaths in 2021, owing to its propensity for distant metastasis [1]. In recent years, the prognosis for metastatic melanoma has dramatically improved with the introduction of immune checkpoint inhibitors (ICIs) and targeted therapies. These advancements have contributed to a nearly 30% reduction in melanoma-related mortality rates in the United States over the past decade [1].

The ICIs enhance the immune response by relieving inhibitory signals in the immune system. They achieve this by directly interacting with immune costimulatory molecules on T cells and within the tumor microenvironment, such as CTLA-4, PD-1, and PDL-1 [2]. Ipilimumab (anti-CTLA-4) was the first ICI utilized in metastatic melanoma, significantly improving overall survival (OS) from 6.4 to 10 months [3]. Similarly, nivolumab (anti-PD-1) further improved progression-free survival (PFS), with less severe immune-related toxicities than ipilimumab [4]. Dual ICI therapy with ipilimumab and nivolumab has demonstrated high efficacy and safety and is currently a first-line strategy in the management of metastatic melanoma [5].

Concurrent with the increasing utilization of ICIs in melanoma, there has been renewed interest in understanding the potential interplay between radiation therapy (RT) and the immune system. One such phenomenon is the abscopal effect, where localized treatments, such as RT, not only shrink the targeted tumor but also induce shrinkage of untreated tumors elsewhere in the body. [6]. The immune correlates of the abscopal effect were notably explored in metastatic melanoma, where a patient receiving ipilimumab monotherapy showed disease progression systemically but experienced a widespread disease response when a single site of metastasis was treated with hypofractionated ablative RT [7]. While precise mechanisms remain elusive, clinical and preclinical models suggest that radiation may increase the number of CD4+ and CD8+ T cells while decreasing the number of myeloid-derived suppressor cells in the tumor microenvironment [7,8]. This hypothesis is supported by the observed timing of the patient’s systemic disease response, which occurred only after a shift from an immune escape phenotype to an immune-mediated tumor elimination phenotype [7].

Although the abscopal effect is highly desired, in practice, it remains an exceedingly rare phenomenon, with limited published data supporting its clinical utility. To that end, a recent meta-analysis of patient-level data showed no clear trend between radiation dose and the use of ICI in eliciting the abscopal effect [6]. Given the relatively low number of reported abscopal effects, we, therefore, aim to share our recent experience with a potent clinical example of this phenomenon. Here, we report a case of an abscopal effect in a patient with metastatic melanoma who was progressing on first-line dual ICI therapy but experienced a rapid and durable systemic response following the administration of hypofractionated palliative RT to a large primary cutaneous melanoma. This case report was de-identified and reviewed by our institutional IRB before publication.

## Case presentation

A 63-year-old female patient presented to urgent care with two large masses on her posterior neck that were painful on palpation. Initial management treated these as infected sebaceous cysts, suspected to be caused by methicillin-resistant *Staphylococcus aureus*, and she was referred to dermatology. The patient completed a course of antibiotics without improvement. A punch biopsy of one of the masses was subsequently performed, and pathology confirmed an invasive, nodular-type melanoma. The histopathology of the mass is shown in Figure 1. Due to the multifocal nature of her cutaneous disease, she underwent a PET/CT scan, which revealed widespread active lesions in the head and neck region, with the largest lesion being the primary melanoma located on the right upper back (3.6 x 2.9 cm; maximum standardized uptake value (SUV_max_) 20.1). There were also level 3 active lymph nodes bilaterally, a right supraclavicular node, and multiple axillary nodal lesions on the right. No other distant metastases were present. Tumor mutational analysis revealed BRAF p.Val600Glu c.1799T>A 50.0%. The tumor mutation burden was 12.0 mutations/Mb and was microsatellite stable. Diagnostic imaging throughout the disease course is shown in Figure 2. 

**Figure 1:** Melanoma histopathology. (A) Portion of the melanoma (20x) that extends to the deep dermis; (B) heavily pigmented cells in the upper dermis (40x); (C, D) large, atypical epithelioid cells throughout the lesion and scattered mitoses (400x).

**Figure 2:** Radiographic response of the primary tumor and satellite nodules. (A) Primary tumor with satellite subcutaneous nodules noted on initial PET/CT scan; (B) CT scan at six months post-RT; (C) CT scan at nine months post-RT; (D) CT scan of the nodules in the right axilla before RT; (E) CT scan of the nodules in the right axilla one month post-RT; (F) CT scan of the nodules in the right axilla three months post-RT; (G) CT scan of the nodules in the right axilla nine months post-RT. The red arrows represent the primary tumor. The green arrows represent the satellite nodules. The yellow arrows represent the nodules specifically in the right axilla. CT: computed tomography, PET: positron emission tomography, RT: radiation therapy.

The patient was started on ipilimumab 3 mg/kg and nivolumab 1 mg/kg for a total of four planned cycles. An interim MRI of the brain ruled out intracranial metastasis. Unfortunately, after the second cycle, worsening of the dominant right upper back mass was noted, with increased size, bleeding, and pain. As a result, the patient was referred by medical oncology for consideration of palliative RT. Following consultation, the treating radiation oncologist recommended a course of hypofractionated palliative RT with 30 Gy in five fractions over 2.5 weeks. A rapid clinical response was noted in the treated primary melanoma on the right upper back (see Figure 3) by the end of the second week of palliative RT. Following RT, a CT of the chest, abdomen, and pelvis was performed and showed an overall decrease in the size of cutaneous nodules and stable to decreased size of axillary adenopathy.

**Figure 3:** Temporal response of the dominant melanoma tumor to hypofractionated RT. (A) Presentation; (B) three weeks post-RT; (C) three months post-RT; (D) four months post-RT. The red arrow represents the primary irradiated melanoma tumor. The green arrows represent nearby unirradiated metastases, which only began to shrink following palliative RT. RT: radiation therapy.

The patient continued nivolumab maintenance at 480 mg every 4 weeks after completing four cycles of dual therapy. A nuclear medicine bone scan was performed five months post-RT and showed no clear active osseous metastases. An additional surveillance CT of the chest, abdomen, and pelvis with contrast showed ongoing systemic disease response, with decreasing right axillary, right chest wall subcutaneous metastasis, cervical lymph nodes, and complete resolution of associated subcutaneous nodules in the nape of the neck. Clinical photos of the nodules on the right and left neck outside the RT field were taken (Figure 3).

## Discussion

​​​​​Here, we present a putative case of an abscopal effect in a patient with metastatic melanoma on dual ICI therapy. The patient experienced clear disease progression while on ICI and only showed systemic improvement in disease burden after hypofractionated RT (HFRT) and local tumor response. The median time for an abscopal response is three months [6], and in our patient, the observed systemic response following local RT was approximately two months. Likewise, although there is no clear trend in the literature regarding the combination of ICI and RT with respect to PFA or OS [6], our patient remains progression-free nearly one year after receiving RT. More broadly, investigators have been frustrated by failed attempts to combine ablative RT techniques with ICIs in clinical trials to improve PFS or OS in patients with advanced tumors, weakening enthusiasm to translate the abscopal effect clinically [9]. Several potential factors may have contributed to the abscopal effect in this case, including the total RT dose administered, the dose per fraction, the melanoma’s relatively high mutational burden, and the concurrent administration of RT with ICI.

The role of radiation fractionation is controversial concerning its potential effect on the immune system and the abscopal effect. Conventional fractionation schedules (those with 1.8-2 Gy/fraction) may negatively affect the ability of immunotherapies to elicit an adequate response [10]. Although there is limited evidence on the optimal dose-fractionation of RT with concurrent ICI, some studies have shown that RT, specifically stereotactic body RT (SBRT), with higher dose-per-fraction (>3 Gy), yields favorable outcomes in metastatic melanoma [10]. A recent meta-analysis found that SBRT may be superior to conventionally fractionated RT (CFRT) approaches involving lower doses per fraction for developing RT-immunotherapy combinations. Additionally, SBRT spares circulating lymphocytes due to its smaller treatment field and fewer dose fractions [8]. Similarly, HFRT has also shown clinical benefit when combined with ICI, with a significantly higher OS (>5 Gy/fraction) [10]. Specifically, HFRT combined with immunotherapy resulted in a three-year OS of 37.3%, compared to 19% with HFRT alone [10]. These findings suggest that radiation dose and fractionation are key factors to investigate for the development of successful RT-immunotherapy combinations.

Similar to the potential effect of fractionation, the total tumor biologic equivalent dose (BED) may also impact immunogenicity following RT. The BED is influenced by the alpha/beta ratio, which measures the intrinsic radiosensitivity of a target tissue, with tumors typically having an alpha/beta ratio of ~10. In an animal model study, a BED of 60 Gy or greater and tumors with a standard alpha/beta ratio of 10 were associated with up to 50% out-of-field responses [11]. Interestingly, higher doses with fewer fractions to surrounding normal tissues increase the risk of late complications in cancer survivors, specifically in gastrointestinal structures and kidneys [11].

Tumor mutational burden (TMB) refers to the number of mutations per DNA megabase and is a biomarker of response to ICI. Melanoma, specifically, is a highly immunogenic tumor with a high mutational burden, as in our case, which explains the efficacy of ICI, such as ipilimumab [12]. A high TMB in melanoma is often considered to be at least 10 mutations/Mb [12]. Our patient’s tumor had a high TMB of 12.0 mutations/Mb. RT also exposes silent immunogenic mutations to the immune system, increasing their presentation by cancer cells [12]. Additionally, RT can increase cancer antigenicity by generating de novo immunogenic mutations [2]. This converts tumors with a low mutational burden into those with a high mutational burden, making the tumors more responsive to ICI [2].

There are increased response and recurrence-free survival rates in melanoma patients with a high TMB and high inflammatory signature who received nivolumab or nivolumab and ipilimumab, compared to patients receiving ipilimumab alone. This was even more pronounced in BRAF wild-type patients compared to those with BRAF mutations [12]. Of note, our patient received a combination of nivolumab and ipilimumab and later continued nivolumab maintenance therapy.

Along with TMB, driver mutations can play a role in immune-mediated responses [12]. BRAF V600E mutations were predominantly found in low-TMB melanoma tumors, whereas KMT2 mutant melanoma was more likely to have a high TMB compared to wild-type tumors. High TMB and BRAF wild-type tumors were associated with prolonged recurrence-free survival and prolonged OS when treated with nivolumab or ipilimumab [12]. Interestingly, our patient had a BRAF V600E mutation but still exhibited a relatively high mutational burden, which contrasts with typical trends.

RT can also have immunosuppressive effects through multiple mechanisms, which may partly explain why the abscopal effect remains a clinically rare phenomenon. One mechanism involves hypoxia-related remodeling of the tumor microenvironment, resulting in the accumulation of immunosuppressive M2-like tumor-associated macrophages, regulatory T cells (Tregs), and exhausted T cells [8]. This remodeling also leads to stromal reactions supported by cancer-associated fibroblast-derived transforming growth factor-B1 and extracellular matrix deposition. Another mechanism involves hypoxia-driven resistance of cancer cells to cytotoxic T lymphocytes, causing downregulation of MHC class I molecules and activation of stress response pathways, such as autophagy. It also leads to lymph node dysfunction and lymphopenia if circulating within the irradiated field [8]. Radiation has also been shown in preclinical models to enhance the generation of Tregs by stimulation of immunomodulatory skin-resident antigen-presenting cells, such as Langerhans cells [13].

## Conclusions

The abscopal effect is a potentially powerful phenomenon that leverages the interplay between RT and immunotherapy. Here, we present a putative case of an abscopal effect in a patient receiving hypofractionated palliative RT. This patient’s clinical benefit from the combination of palliative RT and ipilimumab/nivolumab provides useful perspectives into potential mechanisms by which abscopal RT responses may be elicited and studied in the future. We advocate for more systematic reporting and investigation of the abscopal effect to allow for further understanding of how it may be more effectively harnessed. Additionally, we anticipate future studies incorporating concurrent and adjuvant ICI therapies with RT, which may capitalize on the synergy between these therapies and the abscopal effect to improve patient outcomes.
